# Bioinorganic Synthesis of Polyrhodanine Stabilized Fe_3_O_4_/Graphene Oxide in Microbial Supernatant Media for Anticancer and Antibacterial Applications

**DOI:** 10.1155/2021/9972664

**Published:** 2021-06-25

**Authors:** Seyyed Mojtaba Mousavi, Seyyed Alireza Hashemi, Ahmad Gholami, Navid Omidifar, Maryam Zarei, Sonia Bahrani, Khadije Yousefi, Wei-Hung Chiang, Aziz Babapoor

**Affiliations:** ^1^Department of Chemical Engineering, National Taiwan University of Science and Technology, Taipei, Taiwan; ^2^Nanomaterials and Polymer Nanocomposites Laboratory, School of Engineering, University of British Columbia, Kelowna, BC V1V 1V7, Canada; ^3^Pharmaceutical Sciences Research Center, Shiraz University of Medical Sciences, Shiraz, Iran; ^4^Department of Pathology, School of Medicine, Shiraz University of Medical Sciences, Shiraz, Iran; ^5^Biotechnology Research Center, Shiraz University of Medical Sciences, Shiraz, Iran; ^6^Department of Chemical Engineering, University of Mohaghegh Ardabili (UMA), Ardabil, Iran

## Abstract

Polyrhodanines have been broadly utilized in diverse fields due to their attractive features. The effect of polyrhodanine- (PR-) based materials on human cells can be considered a controversial matter, while many contradictions exist. In this study, we focused on the synthesis of polyrhodanine/Fe_3_O_4_ modified by graphene oxide and the effect of kombucha (Ko) supernatant on results. The general structure of synthetic compounds was determined in detail through Fourier-transform infrared spectroscopy (FT-IR). Also, obtained compounds were morphologically, magnetically, and chemically characterized using scanning electron microscopy (SEM) and vibrating sample magnetometer (VSM), energy dispersive X-ray (EDX) analysis. The antibacterial effects of all synthesized nanomaterials were done according to CLSI against four infamous pathogens. Also, the cytotoxic effects of the synthesized compounds on the human liver cancer cell line (Hep-G2) were assessed by MTT assay. Our results showed that Go/Fe has the highest average inhibitory effect against *Escherichia coli* and *Pseudomonas aeruginosa*, and this compound possesses the least antimicrobial effect on *Staphylococcus aureus*. Considering the viability percent of cells in the PR/GO/Fe_3_O_4_ compound and comparing it with GO/Fe_3_O_4_, it can be understood that the toxic effects of polyrhodanine can diminish the metabolic activity of cells at higher concentrations (mostly more than 50 *µ*g/mL), and PR/Fe_3_O_4_/Ko exhibited some promotive effects on cell growth, which enhanced the viability percent to more than 100%. Similarly, the cell viability percent of PR/GO/Fe_3_O_4_/KO compared to PR/GO/Fe_3_O_4_ is much higher, which can be attributed to the presence of kombucha in the compound. Consequently, based on the results, it can be concluded that this novel polyrhodanine-based nanocompound can act as drug carriers due to their low toxic effects and may open a new window on the antibacterial agents.

## 1. Introduction

Rhodanine monomer is introduced as one of the 4-thiazolidinediones subtypes that can broadly be utilized in pharmaceutical and medical applications [1]. As mentioned in our previous work [2], the rhodanine monomer possesses diverse applicable activities such as antibacterial, antifungal, anti-inflammatory, and antimalarial activities. Due to the outstanding physicochemical properties, polyrhodanines have gained considerable attention during the last years [3]. Free electron pairs can affect the formation of some vital bonds [4]. As proven before [5], many excellent properties of magnetic nanoparticles such as low cytotoxicity, affordable and ecofriendly performance, and favorable biocompatibility made these materials a potent option for a broad range of usages [6]. By exerting a magnetic field, some localize and recycling properties of magnetic nanoparticles can develop for drug delivery systems [7, 8]. Although magnetic nanoparticles possess several advantageous properties, some significant drawbacks can limit their application. Indeed, these barriers are mostly originating from surface oxidation, magnetic aggregation, and a shortage of functional groups. Hence, to eliminate these mentioned barriers, the designing of polymer-coated magnetic nanoparticles is performed in diverse fields. The magnetic nanoparticles can be protected from aggregation and surface oxidation by using a polymer shell. Also, a polymer shell can increase the stability of magnetic nanoparticles and enhance functional groups. So far, diverse synthetic approaches were proposed to promote the magnetic polymer nanoparticle preparation process [9]. However, many of these methods were using costly and toxic reagents in their multistage preparation. These toxic reagents could affect the biological application of magnetic polymer nanoparticles [10, 11]. Thus, the researchers had tried to provide a facile, ecofriendly, and affordable synthetic approach to improve the activity of the magnetic nanoparticles. Graphene oxide (GO) is known as the oxidized shape of graphene, produced through several chemical oxidation techniques [12]. As shown in Figure 1, these valuable substances possess a combinational structure equipped with different oxygen-based functional groups such as carbonyl, epoxy, carboxylic, and hydroxyl [9, 14, 15]. In the last decade, many efforts have been performed to determine the efficiency of GO in clinical studies. Indeed, the researchers used different animal and human cell lines (in vivo and in vitro) to investigate and confirm the toxicity. Moreover, they utilized various methods and tests to evaluate the biocompatibility performance of GO [11, 13, 16, 17].

Consequently, it is claimed that GO in its hybrid structure can provide low toxic effects that this toxicity can be manipulated by combining GO with other materials [9]. In the last ten years, GO/inorganic nanocomposites have raised substantial interests in biomedical application, with mainly significant antibacterial and anticancer potential [18–20]. In this study, we used a media composed of kombucha supernatant to synthesize polyrhodanine/Fe_3_O_4_ modified by graphene oxide to control the cytotoxic effect and increase their antibacterial activity. In the current study, we have reinforced bioinorganic synthesis of the polymeric structure of polyrhodanine (PR) with magnetite nanoparticles (Fe_3_O_4_) and decorated graphene oxide (GO) with Fe_3_O_4_ nanoparticles (GO-Fe_3_O_4_) toward improving the morphology, structural stability, functional groups, and catalytic activity of PR and Fe_3_O_4_. Recently, the inorganic combination of polymers, based on the use of magnetic solid-phase extraction, has attracted more attention [21]. This type of inorganic synthesis gives the nanocomposite numerous biomedical capabilities and can even be used for environmental purposes [22, 23]. The modification step is also boosting the magnetization of PR and makes it a magnetic retrievable polymeric platform. Afterward, the biocompatibility, sensitivity, activity, morphology, and relative active functional groups of PR were boosted upon the introduction of kombucha solvent to the hybrid platform of PR-GO-Fe_3_O_4_ toward detection of DOX in biological fluids. The developed platform was well-characterized, and its performance for detecting DOX within blood was examined and evaluated in detail. Therefore, this investigation was implemented in three separate sections to describe the synthesis, characterization, and cytotoxic study on polyrhodanine/Fe_3_O_4_ modified by graphene oxide and the effect of kombucha supernatant on results.

In the first section, by using the coprecipitation approach, the magnetic nanoparticles were synthesized, and after that, the polymerization of rhodanine was carried out. During the polymerization process, potassium permanganate acted as an oxidant agent, and thus, the polyrhodanine-coated Fe_3_O_4_ nanoparticles (Fe_3_O_4_/PRd) with core/shell structure were produced. GO, which was prepared using the modified Hummer's method, was applied to modify the surface properties of Fe_3_O_4_/PRd. The active role of GO was indicated in characterization tests. At some stages of the above synthesis, instead of deionized water, a solution containing water and kombucha has been used with a ratio of ten to one, respectively. We compared the characterization tests of compounds with and without kombucha to elucidate the biological applications. In the final section of this investigation, the potential cell toxicity of these produced compounds was assessed by MTT assay.

## 2. Experimental

### 2.1. Materials

All of the materials utilized in this investigation like rhodanine monomer (C_3_H_3_NOS_2_) (97%), polyvinylpyrrolidone (PVP), potassium permanganate (KMnO_4_), iron (III) chloride six hydrate (FeCL_3_·6H_2_O), ferrous (ІІ) sulfate heptahydrate (FeSO_4_·7H_2_O), ammonium hydroxide (NH_4_OH), and graphene were purchased from Merck Co. (Germany). Indeed, all these materials were of analytical grade and applied without further purification process. It is necessary to mention that kombucha SCOBY was obtained from the Caucasus Mountains [9]. Deionized water and kombucha solvent were applied all over the experiment.

### 2.2. Polyrhodanine (PR) Synthesis

To prepare the polyrhodanine, we applied the chemical oxidative polymerization technique. In a typical experiment, 50 mL double-distilled, deionized water containing 0.1 g rhodanine monomers was poured into a beaker, and its temperature was fixed at 80°C. After that, 0.05 gr polyvinylpyrrolidone (PVP) was added to the above solution under intensive stirring. For preventing adherence and aggregation of monomers, the solution was put in a cool place. Then, 50 mL double-distilled, deionized water containing 0.5 g KMnO_4_ was added dropwise into the solution at 25°C for 24 hours. To separate the polymers, in the next step, the solution was centrifuged (about 30 min 5000 rpm) and then washed with double-distilled, deionized water and dried at 80°C for 24 h and saved for later experiments.

### 2.3. Preparation of Graphene Oxide-Coated Fe_3_O_4_ Nanoparticles (GO/Fe_3_O_4_)

In this case, 320 mL double-distilled, deionized water was poured into a round-bottom flask, and the temperature was fixed at 80°C. After that, 4.55 g of FeCl_3_·6H_2_O and 3.89 g of FeSO_4_·7H_2_O were added to the mentioned flask and stirred for 90 minutes. Then, 100 mL deionized water was added to 0.0844 g GO, mixed ultrasonically for half an hour, and poured into the previous solution. The obtained solution was mixed at 80°C, and after that, 40 mL NH_3_ was gradually added to the solution mentioned above and stirred for 2 hours. After filtration, the suspension was washed, and the pH scale was set at 7 and finally dried in an oven at 100°C for 60 minutes.

### 2.4. Preparation of Polyrhodanine/GO/Fe_3_O_4_

First, 0.15 g PR was dissolved in 50 mL double-distilled deionized water and was poured into a beaker. Then, along with stirring, 0.5 gr GO/Fe_3_O_4_ was added to the above suspension for 30 minutes. The obtained solution was stirred for half an hour, and after that, 0.25 g KMnO_4_ was dissolved in 50 mL double-distilled, deionized water was added dropwise as an oxidant into the solution under stirring at room temperature for 24 h. After 24 hours, the suspension was filtered and washed simultaneously with deionized water to set the pH on 7 and dried in a vacuum oven for 2 h at 100°C. To produce polyrhodanine/GO/Fe_3_O_4_ based on kombucha solvent (PR/GO/Fe_3_O_4_/Ko) in all stages of the above synthesis, instead of deionized water, a solution containing water and kombucha has been used with a ratio of ten to one, respectively.

### 2.5. Characterization

All synthetic compounds were characterized using Tensor ІІ FT-IR spectroscopy (Bruker, Germany) in the frequency range of 4000–400 cm^−1^. The EDX spectroscopy and morphology of all samples were measured by MRA ІІІ (TESCAN). The magnetization characterization was measured by MDKB VSM (Mdk, Iran) using changing H between +20,000 Oe and −20,000 Oe.

### 2.6. Minimum Inhibitory Concentration (MIC), Minimum Bactericidal Concentration (MBC), and Minimum Fungicidal Concentration (MFC)

The test organisms used in this study were *Pseudomonas aeruginosa* (ATCC 9027)*, Escherichia coli* (ATCC 15224), *Enterococcus faecalis* (ATCC 19433)*, Staphylococcus aureus* (ATCC 29737), and *Candida albicans* (PTCC 5027).

In this regard, several antimicrobial assays including minimum inhibitory concentration (MIC), minimum bactericidal concentration (MBC), and minimum Fungicidal concentration (MFC) were performed. All experiments were performed six times according to the guidelines of the Clinical and Laboratory Standards Institute [24–26].

Briefly, the two-fold serial dilution of compounds from the concentration of 1000 to 7.8 *μ*g/mL was prepared in a 96-well microplate containing Muller-Hinton broth. After separately adding each test microorganism to microplates and after incubation for 24 h, the optical density was read using an ELISA plate reader (BioTek, USA) at 600 nm. MIC was defined when a concentration of compounds (90%) of the bacterial growth was inhibited [27].

For MBC and MFC, all the microorganisms were cultured for 24 hours in BHI; after that, a stock with a 10^5^-10^6^ CFU/mL concentration was prepared for each microorganism. Briefly, to determine the minimum bactericidal concentrations (MBCs), those media from wells that possessed no bacterial growth were cultured on nutrient agar and incubated overnight at 37°C. This experiment was designed for MFC value calculation when the fungal strain was the culture in the RPMI medium. The lowest concentration value of the sample, which causes less than four visible colonies, was considered MBC for all bacterial strains and MFC for fungal strain [28, 29]. These tests were accomplished in triplicate.

### 2.7. In Vitro Cell Toxicity Assay

Cytotoxicity of all the synthetic compounds on the Hep-G2 cell line was assessed using standard MTT colorimetric assay [30, 31]. Six different concentrations of compounds from 1 to 500 *μ*g/mL were chosen. Hep-G2 cells were suspended in Dulbecco's modified Eagle's medium (DMEM) media containing 10% FBS and roughly 1% penicillin and streptomycin. In short, a certain number of Hep-G2 cells (10^4^) were located in each well of the microplate, and also, they were incubated in a humidified atmosphere of 5% CO_2_ and 95% air at 37°C to let the cells stick and reach about 75–90% confluence. On the next day, the media in each well were changed by 100 *μ*L of each compound suspension prepared by DMEM media previously, and therefore, the plates were incubated at the same condition of the last day. After 24 hours, all the medium was removed from the plate, and then all the wells were rinsed with PBS for about three minutes. Finally, 30 *µ*l MTT solution (4 mg/mL in media) [3-(4,5-dimethylthiazol-2-yl)-2,5-diphenyltetrazolium bromide] was injected into each well and incubated again for about 4 hours. It can be said that this assay is mostly based on the enzymatic diminution of MTT in living, metabolically active cells. In this case, after removing the MTT solution and adding 100 *μ*L of dimethyl sulfoxide (DMSO), and incubating for 10 minutes, blue/purple formazan crystals were produced. The plate was shaken in a double orbital manner (for 5 minutes) to completely dissolve formazan crystals. Finally, the optical absorption of the mentioned solution was recorded at 540 nm using an ELISA plate reader (Model 50, Bio-Rad Corp, Hercules, California, USA). All tests were accomplished in triplicate. In this investigation, the wells comprising untreated Hep-G2 cells were regarded as the positive control (100% viability), and also those wells containing culture medium were considered the negative control (0%). The following equation can describe the calculations of cell viability.

(1) $$\begin{array}{c} \%\text{ cell viability}=\frac{\left[\text{OD}\left(\text{cell}+\text{compound}\right)-\text{OD}\left(\text{compound}\right)\right]}{\left[\text{OD}\left(\text{cell}\right)-\text{OD}\left(\text{DMEM}\right)\right]}*100. \end{array}$$

### 2.8. Statistical Analysis

In this study, Statistical Package for the Social Sciences (SPSS) 22.0 software (SPSS Inc., Chicago, IL, USA) was utilized to analyze and inquire about the biological results. For investigating the results of antibacterial and cytotoxicity tests, one-way ANOVA/Tukey tests were applied to analyze any differences in the mean viability percent of the investigations nanoparticles. This experiment was repeated six times, and the significance level was considered at 0.05.

## 3. Results and Discussion

### 3.1. Synthesis and Characterization

In this section, developed nanomaterials were well-characterized using diverse analyses. In Figure 2(a), a view of the FT-IR spectrum of (I) Fe_3_O_4_, (II) GO-Fe_3_O_4_, (III) PR-Fe_3_O_4_, (IV) PR-GO-Fe_3_O_4,_ and (V) modified PR-GO-Fe_3_O_4_ with kombucha solvent can be seen. As shown in part (I), Fe_3_O_4_ is successfully synthesized and presented as a fingerprint of magnetite nanoparticles. In this matter, the peak between regions 530–630 cm^−1^ corresponds to the stretching vibration of the Fe-O functional group related to magnetite nanoparticles. This peak for developed Fe_3_O_4_ appeared at a wavenumber of 543 cm^−1^. Moreover, other peaks within the FT-IR spectrum of Fe_3_O_4_ are attributed to sp^2^ alkene of C-H band related to disubstituted-E (908 cm^−1^), C-H stretching vibration (1094 cm^−1^), FeOO^−^ (1637 cm^−1^), and hydroxyl functional groups (−OH) (3423 cm^−1^). In part (II), the FT-IR spectrum of GO-Fe_3_O_4_ can be seen; in this part, GO is successfully decorated with magnetite nanoparticles. This matter can be confirmed via simultaneous existence of Fe_3_O_4_ fingerprint at 537 cm^−1^ related to Fe-O functional group along with fingerprint of GO at 1637.14 cm^−1^, which is related to unoxidized C=C double bond carbon atoms. Other peaks within this spectrum correspond to C-H sp^2^ alkene (845 cm^−1^), C-O epoxide (1091 cm^−1^), C-H (1429 cm^−1^), and hydroxyl functional groups (3206 cm^−1^). These outcomes justified the formation of magnetite nanoparticles and modified GO with magnetite nanoparticles, which can be used as additives to modify PR-derived materials. In Figure 2(a) (III), the FT-IR spectrum of PR-Fe_3_O_4_ can be seen. As depicted within this spectrum, sharp peaks at 1454 and 1632 cm^−1^ are attributed to the C=N^+^ stretching and C=C stretching vibration of polymeric chains, which confirm the successful fabrication of PR out of rhodanine monomer through the oxidation process. Moreover, the presence of the Fe-O functional group at a wavenumber of 583 cm^−1^ confirms the interaction of magnetite nanoparticles with the polymeric structure of PR. The other appeared peaks within the PR-Fe_3_O_4_ spectrum correspond to the sp^2^ C-H (829 cm^−1^), C-O functional groups (1111 cm^−1^), C-O stretching, vibration (1201 cm^−1^), C=O stretching vibration (1707 cm^−1^), and –OH functional group (3224 cm^−1^). Besides, the FT-IR spectrum of PR-GO-Fe_3_O_4_ can be seen in Figure 2(a) (IV). As illustrated, GO-Fe_3_O_4_ is well-interacted with PR media and formed an integrated polymeric structure; this outcome could be justified via the existence of PR and GO-Fe_3_O_4_-related FT-IR peaks with less intensity. In this matter, appeared vibrations attributed to the Fe-O (546 cm^−1^), sp^2^ C-H (837 cm^−1^), C-O epoxide (1098 cm^−1^), C=N^+^ (1425 cm^−1^), and amine functional groups (1548 cm^−1^) improved the polymeric structure of PR upon increasing the intensity of C=N^+^- and C=C-related peaks. However, it restricted the formation of Fe-O and thus magnetic domain within the polymeric structure of PR. As shown in Figure 2(a) (V), Fe-O-related peak is removed, and C=N^+^- and C=C-related peaks at 1322 and 1618 cm^−1^, respectively, become shaper with more intensity. Additionally, related peaks of C-O epoxide and –OH functional groups appeared at 1063 and 3340 cm^−1^, respectively.  Figure 3(b) shows that the VSM results of GO-Fe_3_O_4_, PR-Fe_3_O_4_, and PR-GO-Fe_3_O_4_ can be seen. As shown, all developed materials exhibiting an S-like curve show their superparamagnetic nature along with superior magnetization (*M*_s_) of about 16.91, 46.76, and 64.54 emu·gr^−1^ for GO-Fe_3_O_4_, PR-Fe_3_O_4,_ and PR-GO-Fe_3_O_4_, respectively. These data showed the potential of advanced materials as ultrasensitive and retrievable biosensors to detect selected targets within biological fluids.

In Figure 3, the outcome of EDX analysis for (a) PR-Fe_3_O_4_, (b) PR-GO-Fe_3_O_4,_ and (c) modified PR-GO-Fe_3_O_4_ with kombucha solvent can be seen, respectively. As shown in part Figure 3(a), PR-Fe_3_O_4_ is successfully synthesized with 23.24/38.31, 4.11/5.81, 36.18/44.76, 0.08/0.05, 4.58/1.65, and 22.60/8.01 w%/A% of carbon, nitrogen, oxygen, sulfur, manganese, and iron, respectively. These data are in well accord with FT-IR and VSM analysis and confirmed the successful fabrication of PR and its integration with magnetite nanoparticles, making it a superparamagnetic polymeric structure. Moreover, in Figure 3(b), EDX analysis of PR-Fe_3_O_4_-GO can be seen. This sample consists of 15.98/23.32, 5.60/7.00, 57.24/62.68, 1.56/0.85, and 19.63/6.16 w%/A% of carbon, nitrogen, oxygen, sulfur, and iron, respectively. Furthermore, the modification of PR-Fe_3_O_4_-GO with kombucha solvent significantly improved its functional groups. However, the ratio of iron has sharply declined, and the final product turned into the bioimproved nonmagnetic polymeric structure. In this regard, modified PR-Fe_3_O_4_-GO with kombucha solvent (Figure 3(c)) showed 18.46/24.44, 6.13/6.95, 65.91/65.48, 1.34/0.66, 0.22/0.09, 1.09/0.43, 6.59/1.88, and 0.26/0.06 of carbon, nitrogen, oxygen, sulfur, potassium, calcium, iron, and zinc, respectively.

Besides, a morphological view of developed polymeric structures can be seen in Figure 4. As shown in Figures 4(a) and 4(b), the primary modified PR with Fe_3_O_4_ showed a more rigid structure with a uniform size distribution, while modification of PR with GO-Fe_3_O_4_ significantly improved the morphology and polymeric structure of the final product (Figures 5(c) and 5(d)). More importantly, according to the obtained data from FT-IR and EDX analyses, modification of PR-GO-Fe_3_O_4_ with kombucha solvent boosted the polymeric structure of PR and increased the related intensity of C=N^+^ and C=C groups of PR. Likewise, the outcome of SEM images of bioenhanced PR-GO-Fe_3_O_4_ showed similar results. The introduction of kombucha solvent to this system furtherly improved the morphology and polymeric structure of PR-GO-Fe_3_O_4,_ enhancing the sensitivity of the final biosensor for accurate detection of target compounds within biological fluids. In addition, a morphological view of developed polymeric structures can be seen in Figure 4. As shown in Figures 5(a) and 5(b), the primary modified PR with Fe_3_O_4_ showed a more rigid structure with a uniform size distribution, while modification of PR with GO-Fe_3_O_4_ significantly improved the morphology and polymeric structure of the final product (Figures 5(c) and 5(d)). More importantly, according to obtained data from FT-IR and EDX analyses, modification of PR-GO-Fe_3_O_4_ with kombucha solvent boosted the polymeric structure of PR and increased the related intensity of C=N^+^ and C=C groups of PR. Likewise, the outcome of SEM images of bioenhanced PR-GO-Fe_3_O_4_ showed similar outcomes. The introduction of kombucha solvent to this system furtherly improved the morphology and polymeric structure of PR-GO-Fe_3_O_4,_ enhancing the sensitivity of the final biosensor for accurate detection of target compounds within biological fluids.

### 3.2. Antimicrobial Studies

In this experiment, the inhibitory effects of PR/Fe, PR/Fe/Go, Go/Fe, PR/Fe/Ko, and PR/Go/Fe/Ko compounds against the four mentioned bacterial strains and a fungus were evaluated through microdilution broth technique [32]. The results are demonstrated in Figure 5.

In high concentrations (i.e., 1000, 500 *µ*g/mL), all the compounds have antibacterial effects against the mentioned microorganisms. It can be stated that, by increasing the concentration value, antibacterial effects grow in a concentration-dependent manner. The obtained results have revealed that the inhibitory effects of compounds against fungus, Gram-negative, and Gram-positive bacterial strains are not similar. Among all agents, Go/Fe has the highest average inhibitory effects against *Escherichia coli* and *Pseudomonas aeruginosa*, and this compound possesses the least antimicrobial effect on *Staphylococcus aureus*. Some primitive bacterial growth activities were obtained in lower concentrations (mostly less than 15.62 *µ*g/mL) for all the compounds, leading to increased viability percentages to more than 100%. At the most diluted concentration of the experiment (7.8 *µ*g/mL), the viability of *Enterococcus faecalis*, *Staphylococcus aureus*, and *Candida albicans* exposed to PR/Fe/KO was 172%, 190%, and 151%, respectively, which demonstrated the most primitive activity. The best primitive effects against *E. coli* were assigned to PR/Fe at 7.8 *µ*g/mL, and *Pseudomonas aeruginosa* showed about 50% growth enhancement being exposed to PR/Fe/Go at 7.8 *µ*g/mL. Based on the results summarized in Table 1, it can be claimed that Go/Fe showed the most inhibitory effect on all mentioned microorganisms among the tested compounds. These results were confirmed by Shaobin Liu who compared the antibacterial activity of four types of graphene-based materials (graphite (Gt), graphite oxide (GtO), graphene oxide (GO), and reduced graphene oxide (rGO)) toward a bacterial model—*Escherichia coli*. Under similar concentration and incubation conditions, GO dispersion shows the highest antibacterial activity, sequentially followed by rGO, Gt, and GtO [33].

Although the antimicrobial effects of GO/Fe nanocomposite have been studied in few studies, many recent studies have examined the antimicrobial effects of GO nanocomposites with other inorganic materials, especially silver nanoparticles [23, 34, 35]. However, it has been repeatedly shown that the antimicrobial effects of magnetic nanoparticles are negligible [28, 36, 37], and the antimicrobial results of this study are comparable to the results of GO/silver nanocomposites. These effects, which are naturally less than GO/silver nanocomposites, could be due to the added effect of natural compounds attached to the nanoparticle surface due to bioinorganic synthesis. Such an additive effect has already been shown in other nanocomposites [20, 24, 26, 30].

A recent study by Zachanowicz et al. found that the number of viable bacteria was significantly reduced after exposure to binary polyrhodanine manganese ferrite nanohybrids. This effect was directly related to the amount of nanohybrid polymer content, and the higher the amount, the more antimicrobial effects [38]. The antibacterial activity of PR/Fe/Go synthesized in kombucha supernatant media showed more potent than their non-bioinorganic synthesis. This antibacterial activity can be applied in the biomedical and environmental fields because in this nanocomposite the PR is an antibacterial part and Fe_3_O_4_ might play a role as a material collector after the disinfection process due to magnetic properties in the environment or human body.

### 3.3. Cytotoxic Study

A common and acceptable approach for the assessment of cell viability is the MTT assay. This method can also detect and determine biomaterial toxicity [20, 39]. MTT assay can depict the metabolism and mitochondrial activity of cells. In this present experiment, we decided the viability or proliferation of hepatocarcinoma (Hep-G2) cells after 24 hours of treatment with synthetic compounds such as Fe, PR/Fe_3_O_4_, PR/GO/Fe_3_O_4_, PR/GO/Fe_3_O_4_/Ko, PR/Fe_3_O_4_/Ko, and GO/Fe_3_O_4_ (Figure 6).

The metabolic performance of cells was changed in a dose-dependent manner by all of the compounds, where the dosage of compounds varied from 1 to 500 *μ*g/mL. As shown in Figure 6, the cytotoxicity of Fe_3_O_4_ was enhanced by enhancing the concentration value. Indeed, by increasing the concentration from 1 to 500 *μ*g/mL, the cell viability percent was diminished from 132% to 88%. It can be stated that Fe_3_O_4_ has no cytotoxic effect on the Hep-G2 cell line [30, 40]. When PR/Fe_3_O_4_ treated the cells with a concentration from 1 to 10 *µ*g/mL, the metabolic activity related to cell viability was more than 100%. However, at 50 *μ*g/mL and higher concentrations, the Hep-G2 cells represented a considerable loss in cell viability of about 44%. Zachanowicz et al. have claimed that pure polyrhodanine has toxic effects in some concentrations [32]. In contrast, it is proven that Fe_3_O_4_ nanoparticles are not harmful, especially in low concentrations comparing the cytotoxic effects of Fe_3_O_4_, PR/Fe_3_O_4_, and PR/GO/Fe_3_O_4_ against Hep-G2 cell line, as shown in Figure 4. PR/GO/Fe_3_O_4_ is more toxic, while the nontoxic effects of Fe_3_O_4_/GO on both animal and human cells were reported previously [20, 41]. After 24 h, PR/GO/Fe_3_O_4_, by increasing the concentration from 1 to 500 *µ*g/mL, the cell viability percent decreased from 112 to approximately 36 because of polyrhodanine. The performance of GO/Fe_3_O_4_ in comparison with other compounds is entirely different. This compound exhibited no toxic effect on Hep-G2 cells, and the viability percent was more than 130%, especially in higher concentrations (100, 200, and 500 *µ*g/mL). The exposed cells and control were assessed by optical microscopy to confirm the biocompatibility or toxicity of the compounds.  Figure 7 shows the general appearance and shape of untreated and treated cells (Hep-G2 cells treated with 50 *μ*g/mL GO/Fe_3_O_4_). In another research, the findings revealed that both bare Fe_3_O_4_ and Fe_3_O_4_-PEG inhibited SKOV-3 cell proliferation, resulting in programmed cell death. Cytotoxic activity against SKOV-3 cells increased with NIR laser irradiation, while AMF induction heating significantly increased cytotoxic activity [42].

## 4. Conclusions

Polyrhodanines have been broadly utilized in diverse fields due to their attractive features. In this study, we focused on the synthesis of polyrhodanine/Fe_3_O_4_ modified by graphene oxide and the effect of kombucha (Ko) supernatant on results. The antibacterial effects of all synthesized nanomaterials were done according to CLSI against four infamous pathogens. Also, the cytotoxic effects of the synthesized compounds on the human liver cancer cell line (Hep-G2) were assessed by MTT assay. Our results showed that Go/Fe has the highest average inhibitory effects against *Escherichia coli* and *Pseudomonas aeruginosa*, and this compound possesses the least antimicrobial effect on *Staphylococcus aureus*. Considering the viability percent of cells in the PR/GO/Fe_3_O_4_ compound and comparing it with GO/Fe_3_O_4_, it can be understood that the toxic effects of polyrhodanine can diminish the metabolic activity of cells at higher concentrations (mostly more than 50 *µ*g/mL), and PR/Fe_3_O_4_/Ko exhibited some promotive effects on cell growth, which enhanced the viability percent to more than 100%. Similarly, the cell viability percent of PR/GO/Fe_3_O_4_/Ko compared to PR/GO/Fe_3_O_4_ is much higher, which can be attributed to the presence of kombucha in the compound.

## Figures and Tables

**Figure 1:** The structure of GO with functional groups [13].

**Figure 2:** (a) FT-IR spectrums of (I) Fe_3_O_4_, (II) GO-Fe_3_O_4_, (III) PR-Fe_3_O_4_, (IV) PR-GO-Fe_3_O_4,_ and (V) modified PR-GO-Fe_3_O_4_ with kombucha solvent; (b) VSM results of GO-Fe_3_O_4_, PR-Fe_3_O_4,_ and PR-GO-Fe_3_O_4_.

**Figure 3:** EDX analysis of (a) PR-Fe_3_O_4_, (b) PR-GO-Fe_3_O_4,_ and (c) modified PR-GO-Fe_3_O_4_ with kombucha solvent.

**Figure 4:** SEM images of ((a), (b)) PR-Fe_3_O_4_, ((c), (d)) PR-GO-Fe_3_O_4_, and ((e), (f)) modified PR-GO-Fe_3_O_4_ with kombucha solvent.

**Figure 5:** The effects of nanocomposite on the antibacterial of different samples. (a) Effect of nanoparticles on *E. coli*. (b) Effect of nanoparticles on *Pseudomonas aeruginosa*. (c) Effect of nanoparticles on *Staphylococcus aureus*. (d) Effect of nanoparticles on *Enterococcus faecalis*. (e) Effect of nanoparticles on *Candida albicans*.

**Figure 6:** Effect of compounds on cell viability of MTT assay for all tested concentrations on Hep-G2 cells after 24 h in comparison with control (untreated cell). Each bar represents the mean ± SD (standard deviation) of three independent tests.

**Figure 7:** Optical microscopy of (a) untreated Hep-G2 cells and (b) Hep-G2 cells treated with 50 *μ*g/mL GO/Fe_3_O_4_.

**Table 1:** MIC and MBC/MFC values of compounds against microorganisms.

Microorganisms		PR/Fe (*µ*g/mL)		PR/Go/Fe (*µ*g/mL)		Go/Fe (*µ*g/mL)		PR/Fe/Ko (*µ*g/mL)		PR/Go/Fe/Ko (*µ*g/mL)	
		MIC	MBC/MFC	MIC	MBC/MFC	MIC	MBC/MFC	MIC	MBC/MFC	MIC	MBC/MFC
Gram-positive strains	*Staphylococcus aureus*	250	>250	1000	1000	125	>250	1000	1000	250	250
	*Enterococcus faecalis*	250	250	250	250	125	125	1000	1000	250	250

Gram-negative strains	*E. coli*	125	250	125	>250	62.5	>125	125	>250	125	>250
	*Pseudomonas aeruginosa*	125	125	125	>250	62.5	>125	125	>250	125	>250

Fungus	*Candida albicans*	250	250	500	500	250	250	1000	1000	500	500

## Data Availability

All data used to support the findings of this study are included within the article.
